The article "Packaging Big Data Visualization Based on Computational Intelligence Information Design" was retracted in 2022. Reason: concerns about the peer review.

# Packaging Big Data Visualization Based on Computational Intelligence Information Design

**DOI:** 10.1155/2022/4558839

**Published:** 2022-04-23

**Authors:** Guangchao Zhang

**Affiliations:** College of Art and Design, Hainan University, Haikou 570228, Hainan, China

## Abstract

A method based on a computational intelligence information model is proposed to study the visualization of large data packages. Since the CAIM algorithm only considers the distribution of the largest number of classes in an interval, it offers an optimization method and simultaneously determines the appropriate stopping conditions to avoid overcrowding. The effectiveness of the improved algorithm has been experimentally proven. Methods of character reduction and weight determination are used to reduce the index and weight, establishing a large packaging information system. Experimental results show that the improved algorithm in this article produces more classification rules than the CAIM algorithm, because the discrete intervals created by the CAIM algorithm are relatively simple, but the classification rules are few, but less than the number of CAIM algorithms. Classification rules are generated by entropy-based sampling algorithms. This can make the classification rules simple and universal, and it is clear that the optimal sampling algorithm is more accurate than the CAIM algorithm.

## 1. Introduction

After entering the information age, people's production and life are surrounded by a wide variety of information, and we are already in an information-explosive society. Information has a profound impact on social life, economic production, scientific and technological development, cultural exchange, and many other areas. Efficient collection, proper processing, and rapid dissemination of information resources are effective tools for solving various social problems. With the rapid development of information design technology and the rapid opening of information consumption channels, people are demanding more and more diversification of forms of communication and communication in information design. Only with proper processing and design can all types of information be delivered seamlessly and made public. After World War II, people entered the age of technology and brought a third industrial revolution, the information revolution. Information technology is the soul of social reform and progress in the 21st century. It not only promotes the development of science and technology, but also accelerates the distribution of social resources. It has developed into the core technology of contemporary society. The emerging electronic information technology has changed people's ways and means of using information. Machines have gradually replaced part of people's mental activities to obtain information more quickly and effectively. These changes have gradually led to changes in social form [1].

In modern times, human society has experienced many technological changes, among which information technology is very revolutionary. The digital wave and the wide application of new technology have changed the inherent form of traditional printing media such as books, newspapers, and periodicals. With the transformation of technical means such as information collection, information storage, information resource processing, and information integration and transmission, new electronic media such as mobile newspaper, electronic journal, and e-book have emerged one after another. In the context of contemporary social informatization, information design comes from it. Its application scope is wider and wider, its function is stronger and stronger, and its forms of expression are constantly renovated. It has gradually penetrated into all aspects of people's life. As an important function of data integration and data sharing platform, it occupies an important position [2]. Nowadays, the click through rate of websites with strong professionalism such as “design online” and “visual China” remains high. However, although the society has a high demand rate for the information platform of packaging design (Figure 1), it is rarely systematically sorted out; various packaging design books emerge one after another, but the quality is not good, the Qin Dynasty is uneven, and the relevant background information is lacking, so it is difficult to provide effective guidance. There are also a lot of researches on various data platforms and website construction, but there is a lack of sharing platforms for inquiry, market research, and learning. The cutting-edge technology of information design has not been applied to provide convenient design services [3].

## 2. Literature Review

Guo and Dong proposed a production quality evaluation model, which evaluates production quality through users' satisfaction with visual design. At the same time, the functional architecture of the model is given. The model is used to solve the quality problem in the process of visual design. Through the detailed study of key technologies such as collaborative quality design of visual design products based on customer satisfaction, production process quality control technology for multivariety and small batch, and comprehensive quality evaluation technology for the whole product life cycle, the quality assurance of the model for the visual design process is verified. Emerging technologies such as Internet and artificial intelligence are also widely used in large-scale personalized product customization [4]. Li et al. proposed a research scheme for mass customization of electronic products, which will combine the traditional foundation and Internet technology to realize large-scale visual design. In addition, visual design oriented mobile applications developed based on Internet technology appear on a large scale in enterprises and have a large scale in academic research [5]. Wang et al. designed a platform system based on unity3d to realize the three-dimensional display of industrial products with visual design. With the help of web technology, the three-dimensional graphics of products are displayed on the web page, which visually meets the needs of users for product visual design [6]. Based on the research of personalized virtual product customization system based on Internet, D Floriani designed and implemented a fully personalized product customization system based on web, which truly realized the visual design mode of “users participate in design and manufacturers are responsible for manufacturing” [7]. Xue et al., from the perspective of mass customization practice of the company, develop mobile applications of Android or IOS and build the business on mobile applications, so as to realize the combination of users and the company through mobile applications and facilitate the implementation of visual design services [8]. Xue et al. take automobile visual design as an example to carry out the application design research of visual design. At the same time, let users participate in the actual production process of automobile through the application interface of mobile terminal, meet users' visual design needs, and let users experience the actual production site [8]. Mengyuan et al. studied the construction of data sharing platform, the complementarity between technology and user needs, and the interaction between data sharing platform and user services [9]. In terms of information design methods, Sun proposed that the current information design has changed from design for professionals to design for the general public [10]. Taking the presentation form of information design and information media as the starting point, Akusok discusses the change of information design and communication mode caused by the change of information carrier by analyzing the impact of communication source, transmission path, communication interaction, and media change on information transmission [11]. In terms of network platform construction, Bolón-Canedo et al. put forward relevant concepts of learning network platform, analyzed the important role of resource platform in learning network platform, and put forward relevant construction strategies [12]. Most of the existing online databases take the web retrieval interface as the main construction technology to provide users with free and public retrieval data. According to the database survey reports in recent years, online databases are growing rapidly, which shows that the advantages of online databases in information resource integration and sharing are gradually recognized. With the continuous development of packaging materials, packaging technology, and packaging design, the demand of packaging practitioners for information is increasing. According to the information resource quantity report released by China Internet Network Information Center, there are relatively many databases related to packaging, such as products, pictures, enterprises, newspapers, and periodicals, while the number of systematic learning and interactive databases is small, and the information resource data platform specially corresponding to the packaging industry has not been established.

Based on current research, this paper proposes an information design approach based on computational intelligence. Since the CAIM algorithm only considers the distribution of the largest number of classes in an interval, it offers an optimization method and simultaneously determines the appropriate stopping conditions to avoid overcrowding. The effectiveness of the improved algorithm has been experimentally proven. Methods of character reduction and weight determination are used to reduce the index and weight, establishing a large packaging information system.

## 3. Design Principle and Technology of Packaging Big Data Information Visualization

### 3.1. Application Principles of Gestalt in Information Visualization Design

#### 3.1.1. Proximity Principle

Under the action of proximity principle, observers will be more inclined to treat objects with adjacent spatial positions as categories with the same attribute. The proximity principle reveals the potential logical relationship between information and data, making the visual effect of data display more neat and clear.

#### 3.1.2. Similarity Principle

Under the action of similarity principle, the similarity degree of object attributes has become the main basis for object grouping. Using the similarity principle can effectively create a visual guidance path with a simple hierarchical structure, as shown in Figure 2. Figure 2 distinguishes the groups of different monthly data through the difference of column bar interval distance and distinguishes the types of column bar colors representing rainfall and evaporation, which simplifies the information scanning process and enables the audience to distinguish the symbol types in quick browsing.

#### 3.1.3. Connection Principle

Under the action of connection principle, when facing multiple objects with different attributes, the observer will first use the basic principle for identification. At this time, if there is a more recognizable element to connect multiple objects, it can provide a more effective mode for image recognition or information reading behavior.

#### 3.1.4. Coherence Principle

In the process of visual information reception, the principle of coherence makes the smooth contour have stronger integrity in the eyes of the observer.

#### 3.1.5. Closure Principle

The closure principle holds that if there is a significant difference between the boundary of the graphic area and the adjacent area, the objects in the area will be recognized as the same category or group.  Figure 3 clearly illustrates this principle.

Although in the three pictures in Figure 3 the spacing and shape between the bars of each picture are the same, the results of the observer's classification are quite different after using different graphic elements for regional division.

### 3.2. Information Visualization Technology Based on Visualization

#### 3.2.1. Text Information Visualization

Text information generally includes three aspects: vocabulary, grammar, and word meaning. Text information visualization is equivalent to optimizing the information again. From the perspective of information content, tag cloud is a simple and commonly used visualization technology. This method first directly extracts the main keywords in the text and arranges and combines them according to the specific order and law. If necessary, different colors and font sizes will be used to highlight the importance of the core information, such as using larger font sizes or brighter colors to reflect the importance of vocabulary. The direct result of text information visualization is to make the audience's acceptance and understanding of information more intuitive and accurate.

#### 3.2.2. Multidimensional Information Visualization

Multidimensional information visualization is an important goal of industry information data visualization. In reality, massive data information generally has multidimensional characteristics. When multidimensional data is abstractly expressed in the form of information, because the information itself cannot be three-dimensional, corresponding technologies are needed to realize better and more humanized interaction between the audience and the information. The commonly used methods of multidimensional data visualization include parallel coordinate diagram, scatter diagram matrix, multidimensional scatter diagram, and other representations [13].

#### 3.2.3. Hierarchical Relationship Visualization

Hierarchical relationship visualization is a common method to represent the content structure of abstract information. Through the hierarchical relationship, we can effectively sort out the data content and transform its abstract relationship into an intuitive and visible data structure. There are two main types of visual hierarchical relationship construction technology, namely, space filling method and nonspace filling method.

### 3.3. Discretization of Continuous Attributes

At present, the rule mining algorithms used for classification or decision-making include decision tree (ID3), rough set, genetic algorithm, and so on. However, most data mining algorithms are only used for discrete samples. For example, when using rough set method for attribute reduction, it is difficult to judge whether a continuous attribute in the sample is useful for classification or decision-making. Although C4 5 as an improved algorithm of ID3 can mine the classification rules of continuous attributes, the algorithm can not guarantee the efficiency and the calculation is complex. The packaging design index data is not necessarily discrete; it can also be said that it is often continuous and disorderly. Therefore, it is necessary to choose an appropriate discrete method to pave the way for the later rule mining.

Most of the data collected from the real world is not suitable for direct application to knowledge learning algorithms. The main reasons are as follows: first, the scale of original data is often very large, and there are some interference information, which is imprecise, inconsistent, and incomplete; second, the attribute types of the original data set are often very complex, including not only discrete attribute space, but also continuous attribute space. If such a data set is not processed and directly used in the later algorithm, the corresponding efficiency and accuracy will not be obtained. In addition, most classification algorithms can only deal with the data set of discrete value attributes.

Discretization of continuous attributes is a part of data preprocessing. According to different attribute value ranges, the attributes of the original data set can be divided into three types: Digital attributes (such as page number, 1, 2, 3, and 4), noun attributes (such as color, red, yellow, and blue), and continuous attributes (such as weight and distance). Both digital attributes and noun attributes belong to discrete attributes. After repeated experimental comparison, it is found that the classification results, whether accuracy or efficiency, are significantly improved by discretizing continuous attributes into discrete attributes and then learning classification. To sum up, the overall objectives of the discrete algorithm should be as follows:

- Create a high-quality sorting scheme to help professionals understand the data more easily (the quality of the sampling scheme can be measured by the CAIR criteria, which will be discussed later).
- The separate circuit produced should improve the accuracy and efficiency of the training algorithm (in the case of the decision tree algorithm, the efficiency is determined by the number of rules and the training time).
- The sampling process should take place as soon as possible. Discretization of continuous attributes is to transform the value space of continuous value attributes into a limited number of cells, use some different symbols or numbers to represent the divided interval, and give each interval a discrete value, and use this discrete value to represent all attribute values between cells. It can also be discretized through machine learning, and sample learning makes the discretization results more objective and reasonable. The essence of the discretization process is to give some partition points to divide the attribute space [14].

The general steps of discretization of continuous attributes are shown in Figure 4.

### 3.4. Main Algorithms for Discretization of Continuous Attributes

#### 3.4.1. Discrete Algorithm Classification

Continuous attribute discretization algorithm has different division.

1. According to whether the interaction between attributes is considered when dividing the number of attribute intervals, it can be divided into dynamic discretization algorithm and static discretization algorithm. Bining algorithm is a static discretization algorithm, which defines a parameter K on each attribute to represent the maximum number of intervals divided during discretization, regardless of the influence of other attributes.
2. According to whether the information of decision attributes is used as a reference in the discretization process, it can be divided into supervised discretization and unsupervised discretization algorithms. The early commonly used equal width and equal frequency discretization algorithms belong to unsupervised discretization algorithms. These two algorithms need to preset the number of discrete intervals, which have a large amount of lost information and low classification accuracy. Supervised discretization algorithm refers to decision information, usually combined with classification algorithm. Discretization algorithm based on information entropy and Chi2 correlation algorithm based on statistical *x*^2^ distribution belong to supervised discretization algorithm.
3. According to whether all instances in the dataset are used for attribute discretization, it can be divided into global and local discretization. The local discretization algorithm uses some examples in the data set to divide the attribute interval, which is generally combined with the dynamic discretization algorithm. The global discretization algorithm uses all examples, which is generally combined with the static discretization algorithm. In terms of accuracy, local discretization algorithm is often better than global discretization algorithm, but the execution efficiency of global discretization algorithm is significantly higher than local discretization algorithm.
4. Top-down discretization algorithm and bottom-up discretization algorithm: The top-down discretization algorithm initializes an interval containing all attribute values, then splits it according to a certain standard, and then cycles until a certain stop condition is met; the bottom-up discretization algorithm takes each attribute value as the interval boundary and merges adjacent intervals iteratively according to a certain standard until a certain stop condition is met. The bottom-up discretization algorithm has two key problems: one is how to select adjacent intervals for merging, and the other is how to set a reasonable stop condition. CAIM algorithm belongs to top-down discretization, which is a discretization algorithm based on the relationship between classes and attributes.

The classification of main discretization algorithms is shown in Figure 5.

#### 3.4.2. Description of Main Discretization Algorithms

Equal width and equal frequency discretization algorithm: equal width discretization algorithm is the simplest and earliest attribute discretization method. The value of attribute is divided into *k* intervals of equal width according to the specified parameters. The parameters are user-defined. When the data distribution is uneven, the effect of this kind of algorithm is very poor. The equal frequency discretization algorithm is also divided into *k* intervals, and the number of samples in the interval is the same. These two algorithms are very intuitive and simple but do not consider the sample distribution [15].

Chi series algorithms: ChiMerge algorithm determines whether to merge intervals by calculating *x*^2^ (i.e., confidence). At the beginning of the algorithm, each attribute value is regarded as an interval point, and *x*^2^ is calculated for each pair of adjacent interval points. The interval points with the smallest value are merged until the smallest *x*^2^ value is greater than the preset threshold. This algorithm can only merge two adjacent intervals at a time, so the discretization speed is slow. Chi2 algorithm dynamically sets the threshold to *x*_*a*_^2^ − *x*^2^ and introduces a new stop condition: inconsistency rate. Mod-Chi2 algorithm proposes that the degree of freedom V is determined by the number of decision classes in the two adjacent intervals of the current interval and proposes to use the approximate accuracy as the stop condition. The extended Chi2 algorithm proposes to dynamically increase the critical value by dividing the threshold by $\sqrt{2}v$. This kind of algorithm is based on statistical theory, but the calculation is complex, and the bottom-up method is usually more complex than the top-down method, because at the beginning, all continuous values of attributes are taken as interval points, and then some interval points are merged and deleted in each step. Discrete scheme D divides the continuous value of attribute F into *n* discrete intervals:

(1) $$\begin{array}{c} D:\left\{\left[\left(e_{0},e_{1}\right],\left(e_{1},e_{2}\right],\ldots ,\left(e_{n-1},e_{n}\right)\right]\right\}. \end{array}$$

Each value in attribute F can only be divided into one interval, as shown in Table 1.

In Table 1, the estimated joint probability that the median value of attribute F falls in interval *D*_*r*_=(*e*_*r*−1_, *e*_*r*_] and belongs to class *C* is calculated as follows:

(2) $$\begin{array}{c} p_{ir}=p\left(C_{i},D_{r}|F\right)=\frac{r_{ir}}{M}. \end{array}$$

The estimated edge attribute *p*_*i*+_ with the median value of attribute *f* belonging to class C and the estimated interval edge probability *p*_+*r*_ falling in interval *D*_*r*_=(*e*_*r*−1_, *e*_*r*_] are calculated as follows:

(3) $$\begin{array}{c} p_{ir}=p\left(C_{i}\right)=\frac{M_{i+}}{M},\\ p_{+r}=p\left(D_{r}|F\right)=\frac{M_{+r}}{M}. \end{array}$$

For the class attribute mutual information expression between class variable C and discrete variable D in the two-dimensional matrix given in Table 1, the definition is as follows:

(4) $$\begin{array}{c} I\left(C,D|F\right)=\sum_{i=1}^{S}\sum_{r=1}^{n}p_{ir}\log_{2}\frac{p_{ir}}{p_{i+}p_{+r}}. \end{array}$$

Similarly, the class attribute information and Shannon Di in a given matrix are defined as follows:

(5) $$\begin{array}{c} INFO\left(C,D|F\right)=\sum_{i=1}^{S}\sum_{r=1}^{n}p_{ir}\log_{2}\frac{p_{+r}}{p_{ir}},\\ H\left(C,D|F\right)=\sum_{i=1}^{S}\sum_{r=1}^{n}p_{ir}\log_{2}\frac{1}{p_{ir}}. \end{array}$$

Based on the above three definitions, CAIR standard is defined as follows:

(6) $$\begin{array}{c} R\left(C,D|F\right)=\frac{I\left(C,D|F\right)}{H\left(C,D|F\right)}. \end{array}$$

#### 3.4.3. CAIM Algorithm Description

CAIM standard is used to measure the dependency between the target class and continuous attributes [16]. It is defined as follows:

(7) $$\begin{array}{c} \text{caim}=\frac{\sum_{r=1}^{n}\max_{r}^{2}/M_{+r}}{n}, \end{array}$$

where *n* is the number of current intervals; max_*r*_ is the maximum number of samples in *r* interval.

When all samples in all intervals belong to the same class, the CAIM value reaches the highest, and then

(8) $$\begin{array}{c} \max_{r}=M_{+r},\\ \text{CAIM}=\frac{M}{n}. \end{array}$$

CAIM standard sums each max_*r*_ in *n* intervals. The square of max_*r*_ is divided by *M*_+*r*_ for two reasons.

Considering the negative impact of the class with the largest number of samples in an interval and the samples belonging to the class on the discrete scheme, the more such samples, the larger the *M*_+*r*_ value and the smaller the CAIM value.

Measure the number of max_*r*_. Since the frequency division coefficient *M*_+*r*_ is often greater than or equal to max_*r*_, there will be no overflow error in the calculation process. In order to prevent overflow, the first calculation is multiplied by max_*r*_

(9) $$\begin{array}{c} \frac{\max_{r}^{2}}{M_{+r}}=\frac{\max_{r}}{M_{+r}}\max_{r}. \end{array}$$

The algorithm tends to be a separate circuit with a small interval. Mi in a two-dimensional matrix is not used because they are the total number of objects in category *i*, and they do not differ in different discrete schemes. The CAIM value can be calculated by scanning the 2D matrix once. The CAIM standard has the same characteristics as the CAIR standard, but experimental results show that the CAIM standard creates a smaller number of intervals and, consequently, a higher correlation.

### 3.5. Improvement of Discretization Algorithm Based on CAIM

#### 3.5.1. Problems of CAIM Algorithm

CAIM algorithm has two disadvantages:

First, CAIM usually produces a simple discrete scheme, with the number of intervals very close to the number of target classes. For example, this document uses the data in Table 2 as a training sample, and Table 3 generates a discrete scheme by CAIM. The data set is divided into three intervals: [0.20,1.00], (1.00,6.00], and (6.00,7.00]. The ideal discrete scheme should be divided into five intervals, which shows that the effect of this discrete scheme is not good. If this discrete data is used in the next learning algorithm, the accuracy will further deteriorate [17].

Second, CAIM only considers the distribution of the largest number of classes in an interval. Such thoughts are sometimes unfounded. Take Table 4 as an example for the I_1_ interval of two data sets, D_31_ and D_32_. Since the CAIM separate formula uses only five samples belonging to the target class C_1_ (excluding C_2_ and two samples, three samples of C_3_) to calculate the CAIM value, the two data sets have different data distributions but calculated CAIM values are the same. Such unreasonable situations also occur when considering CAIR guidelines. The two data sets may have the same CAIM value calculated, even if the CAIR values are different.

#### 3.5.2. CAIM Algorithm Optimization

CAIM algorithm used in this paper has been roughly described in Section 3.2. On the one hand, other algorithms or discrete methods such as equal width and equal frequency do not consider the sample distribution, or Chi2 series algorithms have complex calculation and need to look up the table to compare the confidence range. On the other hand, the bottom-up discretization algorithm is more complex than the top-up discretization algorithm. CAIM algorithm has incomparable advantages over other algorithms in these aspects. However, the problem of CAIM algorithm is also described in detail. It only considers the distribution of the largest number of classes in the interval and does not consider the distribution of other classes. Aiming at this point, this paper improves the CAIM standard as follows:

(10) $$\begin{array}{c} \text{nca}\sum_{i=1}^{S}\sum_{r=1}^{n}\frac{q_{ir}^{2}}{M_{i+}M_{+r}}. \end{array}$$

And

(11) $$\begin{array}{c} \frac{q_{ir}^{2}}{M_{i+}M_{+r}}=\frac{q_{ir}}{M_{i+}}\times \frac{q_{ir}}{M_{+r}}. \end{array}$$

The distribution of each class in *r* interval and in attribute value is measured, respectively.

And the termination condition is set to the interval number less than log_2_(*n*) to prevent too many discrete intervals when there are too many classes.

## 4. Experimental Results and Analysis

The data collection sources of knowledge Atlas of packaging big data mainly include open knowledge base, industry websites, academic papers, Chinese patents, and other external data. At present, the big data knowledge map of the packaging industry includes 10 first-class concepts (enterprises, people, patents, institutions, papers, events, etc.), 21 second-class concepts (collective enterprises, private enterprises, equipment, etc.), 29 third-class concepts (packaging equipment, printing equipment, etc.), and 28 fourth-class concepts (general machinery, plastic products, etc.) [18]. Through the analysis of the collected data, it has been confirmed that there are 20 kinds of relationships between concepts that can be extracted, including geographical relationship, causal relationship, affiliation (management) relationship, branch relationship, cooperation relationship, communication relationship, competition relationship, cross relationship, upstream and downstream relationship, ownership (work) relationship, etc. The data sources and rules will be further confirmed later. According to statistics, there are 1456749 data on the platform (see Table 5). The demo of big data knowledge Atlas of packaging industry integrating the above data successfully passed the test and has successfully realized the functions of rapid query and retrieval of industry information resources and basic visual presentation, such as defining the upstream and downstream relationship of the product chain through the object attribute of the concept, finding the target product, and then building the cooperation relationship by finding its affiliated company.

A glass data package containing 214 samples and 9 conditional properties was selected to 6 classes.

As an example of a second property in a glass sample, the data distribution of this property is shown in Figure 6.

Some data of glass dataset after discretization are shown in Table 6.

The discrete data set samples are randomly divided into two groups, 70% as the training set and the remaining 30% as the test set. Rosetta rough set software is used to process and predict the classification accuracy counted by the algorithm. Select rules with accuracy >0.75 and coverage >0.05. The comparison of classification rules and classification test accuracy is shown in Table 7.

From the results, the improved algorithm produces more classification rules than CAIM algorithm. This is because the discrete interval generated by CAIM algorithm is relatively simple, so there are fewer classification rules. However, the number of classification rules generated by the discretization algorithm based on entropy is less than that of the discretization algorithm based on entropy, which can make the classification rules simple and have better universality. Moreover, the optimized discretization algorithm has obviously higher classification accuracy than CAIM algorithm.

## 5. Conclusion

Behind the information design, the study of big data packaging visualization is a real need to support the packaging industry informatization. The improved algorithms in this article produce more classification rules than the CAIM algorithm. Because the discrete intervals generated by the CAIM algorithm are relatively simple, there are few classification rules, but few classification rules are derived from entropy-based sampling algorithms. It is simple and universal in nature, and it is clear that the optimized sampling algorithm is more accurate than the CAIM algorithm classification. Large-scale packaging imaging based on China's packaging big data knowledge meets the new requirements of production intelligence of packaging service functions, deepens the packaging industry informatization and industrialization, and reduces production costs, and flexible response can be shown, to better meet the needs of the industry.

## Figures and Tables

**Figure 1:** Visualization of computational intelligent packaging.

**Figure 2:** Application example of similarity principle.

**Figure 3:** Application example of closure principle. (a) Regional Division I. (b) Regional Division II. (c) Regional Division III.

**Figure 4:** General process of discretization.

**Figure 5:** Classification of discretization method.

**Figure 6:** Distribution of the second attribute data of glass dataset.

**Table 1:** Two-dimensional matrix of attribute F and discrete scheme D.

Class	Interval [*e*_0_, *e*_1_] … (*e*_*r*−1_, *e*_*r*_] … (*e*_*n*−1_, *e*_*n*_]	Sum of class
*C*_1_	*r*_11_ … *r*_1*r*_ … *r*_1n_	*M*_1+_
…	…	…
*C*_*i*_	*r*_*i*1_ … *r*_*ir*_ … *r*_*i*n_	*M*_*i*+_
…	…	…
*C*_*s*_	*r*_*s*1_ … *r*_*sr*_ … *r*_*s*n_	*M*_*s*+_
Sum of intervals	*M*_+1_ … *M*_+*r*_ … *M*_+*n*_	M

**Table 2:** Data set.

Class	Value
1	0.2
1	0.3
1	0.7
1	6.3
1	6.6
1	7.0
2	1.3
2	1.7
2	2.1
2	5.1
2	5.6
2	5.7
3	3.5
3	4.0
3	4.3
3	4.8

**Table 3:** Data set discretization scheme generated by CAIM.

Class	Interval			Sum
	[0.20,1.00]	(1.00,6.00]	(6.00,7.00]	
1	3	0	3	6
2	0	6	0	6
3	0	4	0	4
Sum	3	10	3	16

**Table 4:** Two data sets with the same CAIM value but different data distribution.

Class	Interval		Sum
	*I*_1_	*I*_2_	
Dataset D_31_:CAIM(*I*_1_) = CAIM(*I*_2_) = 2.5			
*C*_1_	6	5	10
*C*_2_	2	3	5
*C*_3_	2	2	5
Sum	12	12	20
Dataset D_32_:CAIM(*I*_1_) = CAIM(*I*_2_) = 2.5			
*C*_1_	6	5	10
*C*_2_	1	4	5
*C*_3_	1	3	5
Sum	12	12	20

**Table 5:** Existing data statistics of packaging big data knowledge map.

Information content	Quantity information
Number of enterprises	51620
Product quantity	785147
Enterprise attribute	619440
Packaging college	85
Packaging paper	457
Total	1456749

**Table 6:** Partial data of glass dataset after discretization.

Sample	RI	Na	Mg	AI	Si	K	Ca	Ba	Fe	Type
1	4	3	1	2	4	1	2	1	1	1
2	3	1	4	3	3	1	1	1	2	1
3	1	3	2	3	2	2	2	1	1	1
4	3	1	3	2	3	2	1	1	1	1
5	2	2	4	3	2	2	1	1	1	1
6	1	1	4	3	2	2	1	1	2	1
7	2	1	4	2	3	1	1	1	1	1
8	4	3	4	3	2	2	2	1	3	1
9	3	4	3	1	1	2	1	1	1	1
…	…	…	…	…	…	…	…	…	…	…

**Table 7:** Comparison of improved algorithm with CAIM algorithm and other discretization algorithms.

Method used	Entropy-based discretization	CAIM algorithm	This paper presents an optimization algorithm
Classification rule	Generate 78 articles	Generate 32 articles	Produce 37 articles
Classification accuracy	46.9%	61.2%	69.7%

## Data Availability

No data were used to support this study.
